# Impacts of Angelica Polysaccharide on Proliferation and Differentiation of Mesenchymal Stem Cells of Rat Bone Marrow

This article has been retracted.

**DOI:** 10.1155/2022/5277356

**Published:** 2022-01-10

**Authors:** Shimao Yang, Fei Gao, Min Li, Zhennan Gao

**Affiliations:** ^1^Department of Oral and Maxillofacial Surgery, School and Hospital of Stomatology, Cheeloo College of Medicine, Shandong University, No. 44-1 Wenhua Road West, Jinan, Shandong 250012, China; ^2^Shandong Provincial Key Laboratory of Oral Tissue Regeneration, No. 44-1 Wenhua Road West, Jinan, Shandong 250012, China; ^3^Shandong Provincial Engineering Laboratory for Dental Materials and Oral Tissue Regeneration, No. 44-1 Wenhua Road West, Jinan, Shandong 250012, China; ^4^Department of Oral and Maxillofacial Surgery, Jinan Stomatology Hospital, No. 101 Jingliu Road, Jinan, Shandong 250001, China; ^5^Department of Nursing, Jinan Stomatology Hospital, No. 101 Jingliu Road, Jinan, Shandong 250001, China; ^6^Department of Oral and Maxillofacial Surgery, School of Stomatology, Dalian Medical University, No. 9 Lvshunnan Road West, Dalian, Liaoning 116041, China

## Abstract

In literature, antiosteoporotic effects of *Angelica sinensis* root have been confirmed, but the impact of *Angelica sinensis* polysaccharide (ASP) on osteoblastic or adipogenic distinction of BMSCs is limited. This paper aimed to explore the role of ASP on proliferation and differentiation of rat BMSCs. Rat BMSCs were subjected to isolation and identification through flow cytometry. The proliferation of rat BMSCs under ASP was performed by CCK-8 kit. Measures of osteogenesis under different concentrations of ASP were detected by using alizarin red staining for mesenchymal cells differentiation and ALP activity assay to identify ALP activity. Quantitative RT-PCR was selected to identify osteoblastic or adipogenic biomarkers from a genetic perspective. Likewise, we have evaluated measures of indicators of Wnt/*β*-catenin signal. ASP significantly promoted the proliferation, increased osteogenesis, and decreased adipogenesis of rat BMSCs within the limit of 20–60 mg/L in a dose-dependent manner but was suppressed at 80 mg/L. The expression of cyclin D1 and *ß*-catenin showed a considerable rise over the course of ASP induced osteogenesis. Dickkopf 1 (DKK1) suppressed the regulation of rat BMSCs differentiation through the mediation of ASP. We have observed that ASP upregulated the osteogenic but downregulated adipogenic differentiation of BMSCs, and our findings help to contribute to effective solutions for treating bone disorders.

## 1. Introduction

Postmenopausal osteoporosis is one of the frequently reported skeletal disorders. This disorder has reportedly been considered one of the most crucial public health concerns of the ageing population. The main cause of postmenopausal osteoporosis is estrogen deficiency, this estrogen deficiency after menopause is linked with increased apoptosis of osteoblast (bone-forming cell) [1]. These features can lead to increases in the possibility of both osteoclastogenesis and osteoclast, thus resulting in reduced weight of bone and elevated likelihood for osteoporosis [2].

Furthermore, estrogen deficiency can cause increased proinflammatory cytokines production, contrasting the decrease in levels of bone-forming factors [3, 4]. This estrogen deficiency can create a more suitable environment for microbial proliferation and thus lead to an increased risk for infections of the oral cavity, which themselves may have a relationship with the varied bone condition of osteoporosis [5]. These factors create a more prone environment for peri-implantitis of osteoporosis patients, which acts as a major contributing component to success or failure for dental implantation in oral operations since it can decline formation of bone and negatively impact osseointegration around implants. Many previous studies have indicated that the pace of osseointegration surrounding dental implantations shows a considerable reduction in osteoporotic circumstances compared to the usual and more traditionally used methods [6, 7]. Therefore, a better understanding of the avoidance of implant loss by enhancing the success ratio for dental implants and of how to increase osseointegration in postmenopausal osteoporosis patients is urgently needed.

*Angelica sinensis* (AS) root is among the herbs commonly applied for the treatment of patients with different afflictions in China. AS extracts reportedly possess neuroprotective, antioxidant, hepatoprotective, antiosteoarthritis, and antitumour character [8–12]. Recently, it has been identified that the application of AS extracts has antiosteoporotic outcomes as reflected in examinations of ovariectomized rats [13]. Moreover, AS has been noted to possibly promote human bone cell growth and differentiation [14]. As suggested, AS extracts are postulated for possible in vitro inhibition of RANKL-affected osteoclast difference of bone marrow macrophages, which implies that AS has the potential to help prevent bone loss [15].

*Angelica sinensis* polysaccharide (ASP) is separated from the roots of *Angelica sinensis*. It is a biomacromolecule and has attracted a great deal of attention due to its capability to perform different bioactivities, for example, hematopoietic, immunomodulatory, hepatoprotective, and antioxidant activities [16–19]. A recent report has demonstrated that AS has antiosteoporotic effects on ovariectomized rats and could be beneficial for human bone cells to grow and differentiate [13, 14].

As one of the components of AS, the impact of ASP on the osteoblastic and adipogenic difference from mesenchymal stem cells of rat bone marrow, have, perhaps surprisingly, been rarely reported upon. Accordingly, in the present research, we sought to explore the effect that ASP could have upon the dynamics of how rat BMSCs grow and differentiate.

Therefore, in this paper, we have explored the role of ASP on the proliferation and differentiation of rat BMSCs. Rat BMSCs were subjected to isolation and identification through flow cytometry. The proliferation of rat BMSCs under ASP was performed by the CCK-8 kit. Measures of osteogenesis under different concentrations of ASP were detected by using alizarin red staining for mesenchymal cells differentiation and ALP activity assay to identify ALP activity.

The remaining section of the paper along with a brief introduction of every section is provided below. In the subsequent section, the proposed methodology is explained along with various metrics and experimental setup and observation. Experimental results and their observations were presented in Section 3 of the manuscript, which is followed by a comprehensive discussion of the achievements of the proposed study in resolving the aforementioned issue. Finally, concluding remarks are given.

## 2. Proposed Scheme Methodology

### 2.1. Cells Culture

Male Sprague-Dawley (SD) rats aged three months were selected for the separation of BMSCs from bone marrow following methods outlined in previous research [20]. Then, cells were suspended in *α*-MEM growth medium added with 20% FBS and antibiotics, including penicillin 100 U/ml and streptomycin 100 mg/ml. The designed medium was changed every three days and was passaged. The following trials were conducted using the cells from replacements corresponding to passage 3.

### 2.2. Flow Cytometry

We determined how various cell surface marker proteins were expressed, including CD29, CD90, CD34, and CD45, through flow cytometry. Flow cytometry was used to identify and measure of expression for antigens expression specific for BMSCs. Cells were separated using Trypsin-EDTA (0.25%, 3–5 min, 37°C) (Hyclone) and were washed with PBSF, which is made by using 5% FBS in phosphate-buffered saline (PBS). Subsequently, around 10^6^ cells/100 *μ*L were stained by using PE-conjugated monoclonal antibody including anti-rat CD90 and CD45 and anti-rat CD29 and CD34 by FITC conjugated. The concentration of 2 g/mL at 4°C for 30 min was used to execute this process. By using this methodology, the stained cells with FITC-or PE-labeled rat anti-mouse IgG were marked as isotype controls. As negative controls, these cells were incubated without any additions of antibodies. The cells were then subjected to washing twice followed by suspension in 400 *μ*L PBSF. Then, all cells were used for flow cytometry analyses by using a Beckman Coulter Cytomics FC 500 (Beckman coulter, FC500, FL, USA) and were examined with the assistance of FlowJo Software (TreeStar, Ashland, OR, USA).

### 2.3. Drug Preparation

*Angelica sinensis* is dry roots that were procured from Union Hospital and collected from Minxian (Gansu Province, China). The polysaccharide was extracted and purified following methods outlined in previous research [21]. The used percentage of sugar in ASP—MW 72.9 kD was roughly 95.1%, and the component monosaccharides were comprised of arabinose, glucose, and galactose, with the molar ratio being = 1 : 2.5 : 7.5 [21, 22].

### 2.4. Cell Proliferation Assay

The 96-well plates were used for plating of BMSCs passage 3 at a concentration of 2 × 10^4^ cells/mL and 200 *μ*L/well. Following 24 hours of culturing, the medium was substituted with a fresh medium in the presence or absence of ASP (20, 40, 60 or 80 mg/L), separately. To perform cell counting, the Kit-8 (CCK-8) (Dojindo, Japan) was used at 1, 3, 5, and 7 days after the initial applications of treatment with ASP. In short, 10 *μ*L of CCK-8 solution was poured into every single well of the 96-well plates, which were then subjected to incubation for 2 hours in a standardized incubator. Afterwards, we assessed measures of absorbance at 450 nm, and we plotted a growth curve upon the basis of changes in absorbance over time. The CCK-8 assay for every single group was conducted in three identically replicated cultures (in triplicate).

### 2.5. Differentiation of BMSCs

To assess measures of the impact of ASP upon how BMSCs differentiated, 6-well plates were used for cell plating at concentrations of 5 × 10^5^ cells/2 mL/well. After overnight culturing, the medium was substituted with the osteogenic medium, which was either supplemented with or lacked supplementation with ASP (20, 40, 60, or 80 mg/L) separately. The basal medium was used to the made osteogenic medium by adding *ß*-glycerophosphate (10 mmol/L), dexamethasone (10 nmol/L), and ascorbate phosphate (50 mg/L). The replacement of osteogenic medium was performed every 3 days. These cells were obtained to perform alkaline phosphatase (ALP), alizarin red staining, qRT-PCR, and Western blotting assays after 2 weeks after additions. To further explore the effect of Wnt/*β*-catenin signaling, we used Dickkopf 1 (DKK1) which is an inhibitor of the Wnt/*β*-catenin signaling channel and coincubated samples and DKK1 with optical concentrations of ASP during osteogenesis of rat BMSCs. For our positive controls, we used cells that were incubated with Wnt3a.

### 2.6. Alkaline Phosphatase (ALP) Activity Assay

ALP is considered a prominent osteoblast-cell marker. Its levels are indicative of the number of osteoblast cells derived from BMSCs after differentiation. In our study, we assessed ALP activity following methods previously outlined [23]. In short, the obtained cells went through three freeze-thaw cycles, and we assessed ALP activity by using assays and according to the transformation from p-nitrophenol phosphate to p-nitrophenol with ALP. The cell lysates were allowed to react with yellow liquid substrate of ALP for a predetermined and specified period, and absorbance was evaluated at 405 nm wavelength. The percentage of protein was assessed by the Bradford assay of Bio-Rad, Hercules, CA, USA, and measures of activity of ALP were based upon U/mg protein. The ALP activity was performed in 3 different cultures.

### 2.7. Alizarin Red Staining

With regards to Alizarin red staining, the culture medium was discarded, and the testing cells were subjected to three washes with PBS and were then fixated in 4% paraformaldehyde for half an hour or 30 minutes. Following three washes using PBS, testing cells were subjected to staining using alizarin red solution for 20 mins. Then, we rinsed cells with PBS to remove nonspecific staining and then examined samples by using an inverted phase-contrast microscopy technique (Olympus IX71, Olympus Optical Co., Tokyo, Japan). The concentration of mineral nodules was evaluated with the assistance of QUANTITY ONE software (Bio-Rad). This experiment was conducted three times (in triplicate).

### 2.8. Total RNA Isolation by Quantitative Real-Time PCR Technique

Total RNA was subjected to isolation from harvested cells with Trizol Reagent (Invitrogen, New York, NY, USA) following all instructions of the manufacturer. Subsequently, the RNA was subjected to DNase treatment, and cDNA was derived from synthesis using the PrimeScript Reverse Transcriptase kit (Takara Bio Inc., Shiga, Japan). Following RT reaction, cDNA was taken for use as the template to perform quantitative real-time PCR (SYBR Green I, Invitrogen, Carlsbad, CA, USA) in real time for runt-related transcription factor 2 (Runx2), osteocalcin (OCN), peroxisome proliferator-activated receptor *γ*2 (PPAR*γ*2), lipoprotein lipase (LPL), cyclin D1, *ß*-catenin, and glyceraldehyde-3-phosphate dehydrogenase (GAPDH), which was employed an internal control. Each quantitative real-time PCR was performed in triplicate with the assistance of an ABI PRISM 7300 real-time PCR System by using Applied Biosystems, Foster City, CA, USA, and the PCR cycling conditions were aligned to manufacturer specifications. The specifics for primer sets and sequences are presented in Table 1. An assessment was conducted for relative expression measurement of gene-specific products using the 2^−△△*Ct*^ method and for the subsequent normalization to GAPDH housekeeping gene expression controls. Every single value refers to the average values taken from individual and separate experiments performed in triplicate.

### 2.9. Western Blotting Assay

In respect of Western blotting assays, cells were subjected to washing with PBS three times. Next, we used RIPA lysis buffer (1 mM MgCl2, 10 mM Tris-HCl pH 7.4, 1% deoxycholate 1% Triton X-100, and 0.1% SDS) to lyse samples for 30 mins on ice. Subsequently, SDS-polyacrylamide gel electrophoresis was used for the separation of extracted proteins before transfer to Millipore polyvinylidene difluoride membrane. Obstruction was caused in these Millipore membranes with BSA 3% by using 0.05% Tris buffer saline- (TBS-) Tween 20 for 2 hours at room temperature, before incubation with anti-cyclin D1 and anti-*β*-catenin, and anti-GAPDH (primary antibodies) for 2 hours at room temperature. Subsequently, to being washed with 0.05% TBS-Tween 20 for three times, membranes were then subjected to incubation with secondary antibody peroxidase-conjugated for 2 hours at room temperature. An enhanced chemiluminescence kit (Millipore) was employed for the reactive bands to be visually presented and assessed. The concentrations for bands were assessed with the Chemi-Doc XRS Gel documentation system and Bio-Rad QUANTITY ONE Software.

### 2.10. Statistical Analysis

SPSS Software version 17.0 (SPSS Inc., Chicago, IL, USA) was used to perform all statistical analysis of paper. Measures for statistics that we used equated the mean ± standard deviation (SD). We compared mean values for experimental samples and those from the control group by using Student's *t*-tests (for two groups). Differences were considered as significant at *p* values of <0.05.

## 3. Experimental Results and Observations

In this section, a detailed comparative analysis of the proposed mechanism, that is, Impacts of Angelica Polysaccharide on Proliferation and Differentiation of Mesenchymal Stem Cells of Rat Bone Marrow, is presented. The performance of the proposed scheme is verified through various parameters, such as flow cytometry, cell growth curves, ALP activity assay, and alizarin red staining. Each of these measures and the proposed scheme performance is presented in both textual and graphical formats.

### 3.1. Flow Cytometry Analysis

As indicated by the outcomes, rat BMSCs of passage 3 involved in this research and surface markers of CD29 and CD90 were reportedly positive but were found to have been negative in CD45 and CD34. The CD45 and CD34 were the cell surface markers bearing linkage with lymphohematopoietic cells Figure 1).

### 3.2. CCK-8 Assay

Cell growth curves over a week of culturing in the absence, or presence, of ASP (20, 40, 60 or 80 mg/L) treatments are shown in Figure 2. On the first day of culture, the growth rate failed to exhibit any noticeable or significant differences among comparisons between all treatment groups (*p* > 0.05). Between day 3 and day 7, greater OD values were observed in the groups subjected to ASP treatments (20, 40, and 60 mg/L) compared to results for the control group (*p* < 0.05). As the concentration of ASP rose from 20 mg/L to 60 mg/L, we found that measures of improvements of cell growth were more noticeable. Nevertheless, cell growth exhibited no improvement at a density of 80 mg/L, which suggested that ASP was conducive to the growth of rat BMSCs in both a dose- and a time-dependent manner within the limits of 20–60 mg/L we assessed in our research approach.

### 3.3. ALP Activity Assay

ALP represents a cell marker of osteoblasts, and its activity is frequently referenced as an important measure that can be used to help demonstrate osteogenesis. For the impact of ASP on osteogenic differentiation of rat BMSCs to be determined, ALP activity was measured. As revealed by the outcomes, ALP activities in ASP treated groups (20, 40, and 60 mg/L) were considerably greater than what was found in the control (*p* < 0.05; Figure 3). Nevertheless, cells treated with 80 mg/L failed to show any enhancement of ALP activity and did not demonstrate any notable differences relative to the control (*p* > 0.05).

### 3.4. Alizarin Red Staining

To assess potential differences induced by ASP to osteogenesis, calcium deposition or calcium content in the cultures was investigated following ASP treatment. Light micrograph images were taken of culture wells containing control cells or containing ASP treated cells stained red, which allowed us to visualize calcium content qualitatively. All cultures exhibited calcium deposition to some degree as the intensity of red staining was found to differ among treatments. ASP treated cells showed a noticeable rise in calcium deposition, which was observed to be dependent upon dosages within the limits of 20–60 mg/L of ASP (Figure 4(a)). Nevertheless, cells subjected to treatment with 80 mg/L demonstrated nearly identical calcium content relative to the control. Moreover, the difference was insignificant between values for control samples and samples treated with 80 mg/L of ASP treated cells (*p* > 0.05). The alizarin red-positive nodules in different cultures were quantified to help assess and support such observation and were performed in triplicate (Figure 4(b)).

### 3.5. Quantitative RT PCR

The quantitative real-time PCRs were conducted to explore how the specific osteoblastic and adipogenic markers, Runx2, OCN, PPAR*γ*2, and LPL, were expressed. The outcomes demonstrated that Runx2 and OCN genes experienced upregulation with ASP treatment (20–60 mg/L). Further, this upregulation showed dosage-dependence within the limit of 20–60 mg/L ASP (*p* < 0.05; Figure 5). Conforming to the prior outcomes in the ALP activity and calcium deposition, the upregulation of the osteoblastic genes was found to have been suppressed at a density of 80 mg/L, and no significant differences were observed between treatments with 80 mg/L ASP treated cells and control cells (*p* > 0.05). Furthermore, we also assessed how adipogenic markers were expressed, including PPAR*γ*2 and LPL. The relative measures of expression of adipogenic genes were opposite to patterns of expression for osteogenic genes (Figure 5(b)). These results conformed to findings from other similarly oriented studies conducted in the past.

### 3.6. Wnt/*β*-Catenin Signaling Assay

The Wnt/*β*-catenin signaling channels reportedly bear an association with dynamics underlying the mechanisms, which influence how osteogenesis is regulated. For a better understanding of the potential impacts of improving osteogenesis by application of ASP, we investigated measures for the assessment of the Wnt/*β*-catenin signaling channels. Quantitative real-time PCR outcomes revealed that the levels of two important Wnt/*β*-catenin signaling genes, *ß*-catenin, and cyclin D1 underwent upregulation when treated with ASP (20–60 mg/L; *p* < 0.05) and further revealed that such upregulation was significant, whereas it indicated that there was no apparent upregulation of such genes when cells were treated with 80 mg/L ASP (*p* > 0.05; Figure 6).

To further explore the effect of Wnt/*β*-catenin signaling, we used Dickkopf 1 (DKK1) which is a known inhibitor of the Wnt/*β*-catenin signaling channel and coincubated samples with this inhibitor and 60 mg/L of ASP during osteogenesis of rat BMSCs. Our results indicated that measures of calcium content showed a clear reduction over the course of cotreatments with DKK1 and 60 mg/L of ASP (Figure 7(a)). Quantification of alizarin red-positive nodules (Figure 7(b)) and ALP activity assay (Figure 8) in various cultures also confirmed similar observations from 3 separate experiments. Also, quantitative real-time PCR results indicated that the cotreatment with DKK1 and 60 mg/L of ASP decreased the measures of expression of Runx2 and OCN, compared to treatments with 60 mg/L of ASP group and compared to results for the Wnt3a treatment group (Figure 9(a)). In contrast, measures of the levels of expression of PPAR*γ*2 and LPL in the 60 mg/L ASP and Wnt3a treatment groups were found to have been lower than what was observed in the control group and the 60 mg/L of ASP + DKK1 treatment group (Figure 9(b)). Further Western blotting assays indicated that the levels of expression of *ß*-catenin and cyclin D1 proteins were inhibited in the DKK1 and 60 mg/L ASP cotreatment group (Figure 10). In this case, we speculate that Wnt/*β*-catenin signaling played a crucial role in improving osteogenesis of rat BMSCs by way of the application of ASP, and we postulate that ASP improved osteogenesis of rat BMSCs by way of upregulating Wnt/*β*-catenin signaling.

## 4. Discussion

As one of the herbs extensively applied in China, AS root reportedly possesses neuroprotection, hepatoprotection, antioxidative, antiosteoarthritis, and antitumour qualities. Recently, AS has been recognized as important as AS extracts have antiosteoporotic properties and have been used to help improve treatment outcomes for ovariectomized rats. ASP, which is a biomacromolecule separated from the roots of AS. ASP has recently been identified for use in helping to improve hypoglycemic and hypolipidemic outcomes by way of assessment in a mouse model using type 2 diabetic mice, and this action was subjected to mediation by having the effects of raising glycogen levels and having induced declines in inflammation-related factors. Recent reports have demonstrated that AS has antiosteoporotic effects on ovariectomized rats and that its use could be beneficial for inducing human bone cells to grow and differentiate positively [13, 14]. However, the impact of ASP on the differentiation of osteoblastic and adipogenic from bone marrow mesenchymal stem cells (BMSCs) of rats has previously been rarely reported upon. Therefore, we sought to investigate the impact of ASP and how its application might induce rat BMSCs to grow and differentiate, and we hoped our investigations would have the potential to contribute new solutions for treating osteoporosis, in particular for improving measures of osseointegration near implantations under osteoporosis.

In our experiments, we have investigated the impacts of ASP and how this might influence rat BMSCs to grow and differentiate. ASP was found to have promoted the proliferation of BMSCs in a way that indicated dependence on time and dosage within the limits of 20–60 mg/L that we tested. In contrast, our results also indicated that this degree of enhancement was failed to be discovered at the levels of 80 mg/L ASP applications. The progression of osteogenesis can be divided into three primary phases including the osteoprogenitor phase, the preosteoblast phase, and the mature osteoblast phase [24]. As an early-stage biomarker for the expectation that osteoblastic cells will differentiate, ALP modulates organic or inorganic phosphate metabolism by way of hydrolyzing phosphate esters and thus plays a crucial role in the transport of materials across plasma membranes, especially for inorganic phosphates [25]. In this study, we found that upregulated ALP activity via ASP (20–60 mg/L) indicated that osteogenesis of rat BMSCs was improved due to the application of ASP. However, we also found that a level of 80 mg/L of ASP did not accelerate ALP activity of BMSCs, and we found that there were no significant differences in measures for this treatment compared to the control treatment (without ASP). Consistently, such results were confirmed by assessments of measures of calcium deposition.

Runx2 is a significant transcription factor influencing the dynamics of osteoblastic differentiation of BMSCs [26]. Runx2 affects how downstream genes maintain osteoblastic phenotypes and how the phenotypes are expressed, for example, in regard to OCN. In this study, we found enhanced expression of Runx2 and OCN, which was an evidence that supported the beneficial effect of ASP treatments from 20 to 60 mg/L on osteoblastic differentiation of BMSCs. As has been shown in previous research, increased levels of bone resorption and decreased bone formation are both significant contributors and role players in the progression of osteoporosis. Nevertheless, in addition to excessive resorption of bone, the additional noteworthy phenomenon that influences the decline of bone volume coincides with the expansion of adipose tissue, and this has often been discovered in osteoporotic patients' bone marrow stroma [27]. This suggests that there should be increased significance attached to adipogenesis in assessments of the dynamics underlying bone loss [28] and that osteoblasts and adipocytes share an inverse relationship, whereby increased osteoblastic differentiation is accompanied by decreased adipocytic differentiation. Similar results with respect to the effects of ASP (20–60 mg/L) upon differentiation of osteogenic and adipogenic BMSCs were found in our research; however, high levels of ASP densities (80 mg/L) had no significant effects.

In recent decades, Wnt signaling has been identified to play a significant role in the fate of cells including cell determination, growth, and differentiation [29, 30]. Canonical Wnt signaling has important impacts on bone weight and has been demonstrated in both animal-based and human-based modelling and patient assessments. A direct role has been identified to be played by *ß*-catenin with respect to the regulation of osteoblast and osteoclast activity, which has been confirmed through empirical research multiple times [31]. For example, in an assessment of mesenchymal osteoblastic precursors, researchers found that *ß*-catenin deficiencies induced a halting of osteoblast progression and embryonic skeletal flaws [32–34]. In our experiments, we found that mechanistic assessments indicated that Wnt/*β*-catenin signaling underwent upregulation throughout the improvement of osteogenesis by applications of ASP (20–60 mg/L), which was correspondingly reflected by way of upregulation of the two critical Wnt/*β*-catenin signaling regulators cyclin D1 and *ß*-catenin. However, such enhancement of osteogenesis showed a substantial reduction when we applied ASP at a concentration of 80 mg/L of ASP. To further explore measures of the effectivity of signaling of Wnt/*β*-catenin, we used Dickkopf 1-DKK1, due to its inhibition properties of the Wnt/*β*-catenin signaling channel. We coincubated samples with DKK1 and ASP (60 mg/L) and measured effects using optical concentrations from samples taken at predetermined time steps during osteogenesis of rat BMSCs. The results indicated that the calcium content was considerably decreased during the cotreatment with DKK1 and 60 mg/L of ASP. Quantification of alizarin red-positive nodules and ALP activity assays in different cultures also provided similar results. Quantitative real-time PCR results demonstrated that the cotreatment with DKK1 and 60 mg/L of ASP decreased the levels of expression of Runx2 and OCN when compared to treatments with only 60 mg/L ASP and when compared to results for the Wnt3a treatment group. Western blotting assays identified that the levels of expression of proteins of *ß*-catenin and cyclin D1 were inhibited in the cotreatment assessment with both DKK1 and 60 mg/L of ASP.

## 5. Conclusion and Future Directive

The experiments, which were carried out during the proposed setup, have confirmed that ASP enhanced the proliferation of rat BMSCs by using dose-dependent methodology within the limit of 20–60 mg/L, whereas this impact was found to have been reduced at concentrations of 80 mg/L. ASP improved indicators for osteoblastic assessments but also suppressed adipocytic differentiation of rat BMSCs in a dose-dependent process. At a concentration of 80 mg/L, we identified that ASP had no statistically significant effect on measures of the differentiation of rat BMSCs. Our findings also indicated that ASP promoted osteogenesis of rat BMSCs by way of upregulating the signaling pathway of Wnt/*β*-catenin. Our novel findings and the potential from results indicating this enhancement will help to contribute to increasingly effective solutions for treating bone disorders.

In future, we are interested to enhance our analysis to other BMCS and to further improve the effectiveness of the proposed study.

## Figures and Tables

**Figure 1:** Results of BMSCs identification with flow cytometry. Note: tested cells: for CD29 and CD90 immunopositive and for CD34 and CD45 immunonegative.

**Figure 2:** CCK-8 assay of rat BMSCs cultured with or without ASP (20 mg/L, 40 mg/L, 60 mg/L, and 80 mg/L) up to 7 days; data were presented as mean ± SD, and SD was indicated by error bars; representation of *p* < 0.05 for 20 mg/LASP versus control. b represents *p* < 0.05 for 40 mg/LASP vs. control, and c represents *p* < 0.05 for 60 mg/LASP versus control.

**Figure 3:** ALP activity assay of rat BMSCs in osteogenic medium after different concentrations of ASP treatment (20 mg/L, 40 mg/L, 60 mg/L, and 80 mg/L). Data were expressed as mean ± SD; error bars were indicated for SD; ^*∗*^*p* < 0.05  versus control, and ^*∗∗*^*p* < 0.01 versus control.

**Figure 4:** Alizarin red staining. (a) Mineral nodule formation in different groups (white arrows). (b) Quantitative results of the mineral nodules.

**Figure 5:** Quantitative real-time PCR results of relative expression levels of Runx2 and OCN (a) and PPAR*γ*2 and LPL (b).

**Figure 6:** Quantitative real-time PCR results of relative expression levels of *ß*-catenin and cyclin D1.

**Figure 7:** Alizarin red staining.

**Figure 8:** Quantitative results of ALP activity assay of rat BMSCs in osteogenic medium after 40 mg/LASP, 40 mg/LASP + DKK1, and Wnt3a treatment, respectively.

**Figure 9:** Quantitative real-time PCR results of relative expression levels of Runx2 and OCN (a) and PPAR*γ*2 and LPL (b).

**Figure 10:** Results of western blot assay of *ß*-catenin and cyclin D1 in different groups.

**Table 1:** Gene-specific primers for real time RT-PCR.

Identified gene	Gene-specific forward primer	Gene-specific reverse primer
Runx2	CGCCTCACAAACAACCACAG	AATGACTCGGTTGGTCTCGG
OCN	GGTGGTGAATAGACTCCGGC	GCAACACATGCCCTAAACGG
PPAR*γ*2	GAGTAGCCTGGGCTGCTTTT	CTGATCACCAGCAGAGGTCC
LPL	TCTGCCCCTTGTAGCTGTTC	TCCGCGTTGCAAAGGGTT
*β*-Catenin	GGCAACCAAGAAAGCAAG	CTGAACAAGAGTCCCAAGGAG
Cyclin D1	D1CCCTCGGTGTCCTACTTCA	GTTTGTTCTCCTCCGCCTCT
GAPDH	TCCATGACAACTTTGGTATCG	TGTAGCCAAATTCGTTGTCA

## Data Availability

We did not obtain analytical permission from the data provider because of trade confidentiality.
